# Single Shot Multibox Detector Automatic Polyp Detection Network Based on Gastrointestinal Endoscopic Images

**DOI:** 10.1155/2021/2144472

**Published:** 2021-11-05

**Authors:** Xiaoling Chen, Kuiling Zhang, Shuying Lin, Kai Feng Dai, Yang Yun

**Affiliations:** ^1^Department of Gastroenterology, Quanzhou First Hospital Affiliated to Fujian Medical University, Quanzhou, Fujian 362000, China; ^2^Department of Endoscope Room, Quanzhou First Hospital Affiliated to Fujian Medical University, Quanzhou, Fujian 362000, China; ^3^Imaging Department, Quanzhou First Hospital Affiliated to Fujian Medical University, Quanzhou, Fujian 362000, China; ^4^Department of Health Medicine, Joint Service Support Force 910 Hospital, Quanzhou, Fujian 362000, China

## Abstract

**Purpose:**

In order to resolve the situation of high missed diagnosis rate and high misdiagnosis rate of the pathological analysis of the gastrointestinal endoscopic images by experts, we propose an automatic polyp detection algorithm based on Single Shot Multibox Detector (SSD).

**Method:**

In the paper, SSD is based on VGG-16, the fully connected layer is changed to a convolutional layer, and four convolutional layers with successively decreasing scales are added as a new network structure. In order to verify the practicability, it is not only compared with manual polyp detection but also with Mask R-CNN.

**Results:**

Multiple experimental results show that the mean Average Precision (mAP) of the SSD network is 95.74%, which is 12.4% higher than the manual detection and 5.7% higher than the Mask R-CNN. When detecting a single frame of image, the detection speed of SSD is 8.41 times that of manual detection.

**Conclusion:**

Based on the traditional pattern recognition algorithm and the target detection algorithm using deep learning, we select a variety of algorithms to identify and classify polyps to achieve efficient detection results. Our research demonstrates that deep learning has a lot of room for development in the field of gastrointestinal image recognition.

## 1. Introduction

Endoscope technology is widely used in the diagnosis of gastrointestinal diseases [1–3]. However, a large number of medical images will be generated during the detection process. It is a very time-consuming and laborious task to only rely on the doctor's naked eyes to identify the lesion-containing part from the large number of gastrointestinal endoscopic images [4–7], and the diagnosis process mainly relies on the doctor's experience and pathology. The diversity of features and the complexity of the gastrointestinal environment and the rate of misdetection and missed detection of lesions are still high, so it is particularly important to develop efficient and accurate endoscopic image lesion detection methods.

The rapid development of medical equipment has promoted the improvement of medical standards to a certain extent and provided guarantee for the timely treatment of the majority of patients. However, each endoscopy will produce a large number of images, and most of them do not contain lesion information. Therefore, before making a diagnosis, clinicians need to spend a lot of energy and time to find images containing lesions from a huge image data set, which increases the workload of doctors. Therefore, it is very necessary to help doctors quickly find and diagnose early lesions, improve doctors' work efficiency, and solve patients' problems in a timely manner. Accurate detection of lesions in medical images provides a guarantee of diagnostic information for clinical applications. This topic is useful for assisting doctors in screening. Diagnosing lesions has important theoretical significance and application value.

In recent years, with the rise of machine learning and artificial intelligence, computer vision has also been further developed. Computer vision mainly uses a computer to simulate people to perform related processing on images and obtain valuable information in pictures. Computer vision has been widely used in many fields such as medical image processing, industrial robots, image monitoring, and unmanned driving, and the effect is also very significant. Target detection is a basic field in computer vision applications. Target detection mainly combines target segmentation and target recognition. Its recognition accuracy, recognition efficiency, and positioning accuracy are the main performance indicators of the entire system. In recent years, with the annual PASCAL VOC challenge [8], more and more teams have participated. Each year, the participating teams propose some advanced algorithms or propose improvements on existing algorithms. It is precisely because of their efforts that target detection has developed rapidly.

With the rise of machine learning, artificial intelligence, and deep learning, many institutions and many colleges and universities have carried out a lot of exploratory work. In 2014, Girshick et al. proposed a deep learning target detection algorithm RCNN [9] based on a region of interest [10] combined with a convolutional neural network (CNN) [11–13], which made a breakthrough in target detection. It has also inspired a large number of outstanding talents to study the target detection algorithm based on deep learning.

The current target detection algorithms based on deep learning are roughly divided into deep learning target detection algorithms based on regions of interest and deep learning target detection algorithms based on regression. Among them, deep learning target detection algorithms based on regions of interest include RCNN [14, 15], SPP-net [16, 17], Fast RCNN [18, 19], Faster RCNN [20, 21], Mask R-CNN [22–25], and YOLO [26, 27].

Gastric polyps have many effects on the stomach. For example, if gastric polyps grow in the cardia, it may cause difficulty in swallowing, because the position of gastric polyps affects normal swallowing ability. If polyps grow in the antrum of the stomach, which is commonly referred to as the pylorus, problems such as pyloric obstruction will easily occur, which will affect the postmeal state. Patients may experience bloating after meals, and in more severe cases, symptoms such as nausea and vomiting may occur. Some patients do not deal with it in time when gastric polyps appear, and eventually they may become cancerous and become gastric cancer.

In order to break the situation of high missed diagnosis rate and high misdiagnosis rate of the pathological part of the gastrointestinal endoscopy image recognized by experts with naked eyes, we propose an algorithm for automatic polyp detection based on SSD [28]. Our purpose is to help doctors quickly find and diagnose early lesions, improve doctors' work efficiency, and solve patients' problems in a timely manner.

## 2. Mythology

### 2.1. Deep Learning

#### 2.1.1. Detection Framework

The polyp detection process based on deep learning algorithm is shown in Figure 1. In the first step, in order to select a clearer lesion-containing image from the endoscopy and construct a data set, preprocessing is required. The preprocessing mainly includes random adjustment of the original image, lesion marking, and data format conversion. The second is to build two deep learning algorithm network models. Model building is an important part of the entire process. The choice of algorithm will directly affect the results of lesion detection. Next, train the sample set and export the training model. Finally, the obtained model is applied to the test set for detection, and the performance of the algorithm model is compared by evaluating the accuracy and detection speed.

#### 2.1.2. SDD Network Structure

Single Shot MultiBox Detector (SDD) is a 2016 ICCV paper. It is the main target detection algorithm so far. SSD is based on a forward propagation CNN network, which generates a series of fixed-size bounding boxes, and the possibility of object instances contained in each box, namely, score. After that, perform a nonmaximum suppression to get the final predictions. The SSD network structure can be seen from the figure divided into two parts: basic network + pyramid network. The basic network is the first 4 layers of VGG-16. The pyramid network is a simple convolutional network that gradually becomes smaller in feature maps and consists of 5 parts. The network structure of SSD is shown as in Figure 2.

#### 2.1.3. Mask R-CNN

The Mask R-CNN network structure is designed on the basis of Faster R-CNN to achieve target detection. The feature extraction backbone network of VGG16 is replaced with Res Net-FPN; the pixel of the feature map and the candidate area cannot be aligned due to the rounding operation. The ROI Pooling layer is replaced by the ROI Align layer; adding an FCN branch to achieve semantic segmentation at the same time has shown excellent results in many large public data sets. The structure of the Mask R-CNN algorithm is shown in Figure 3.

### 2.2. Experimental Treatment

#### 2.2.1. Build a Data Set

In this paper, a total of 4900 gastrointestinal endoscopy images are used for experiments. Two types of lesion images are constructed at the same ratio. The total training set is 2000, and the total verification set is 1500. The test set is divided into images with lesions and normal images without lesions, a total of 1400 open. The specific data division is shown in Table 1.

#### 2.2.2. Image Preprocessing

Image preprocessing is an indispensable link before model training and learning. The purpose is to remove the interference information that is not conducive to model training in the original gastrointestinal endoscopy image, highlight the characteristic information of the included lesions, and improve the efficiency of training and learning. The preprocessing process of this article mainly includes three parts, random adjustment of the original image, lesion marking, and data format conversion.

### 2.3. Evaluation Index

Mean Average Precision (mAP) is a performance metric for this type of algorithm that predicts the target location and category. mAP is very useful for evaluating target localization models, target detection models, and instance segmentation models.

## 3. Results

### 3.1. Data Set Experimental Results

#### 3.1.1. The Impact of Data Set Categories

We, respectively, performed 6000 iterations of Train, Eval, and Test in the esophageal cancer image data set and the mAP (%) of the SDD algorithm and Mask R-CNN algorithm on the image test set. The detection results are shown in Figure 4.

It can be seen from Figure 4 that comparing the SDD algorithm and the Mask R-CNN algorithm, the mAP of the training verification sample set Test on the esophageal cancer image test set is higher than the training sample set Train and Eval.

#### 3.1.2. The Influence of the Number of Iterations

When we iterate 3000, 6000, 9000, and 12000 times on the image training verification sample set Test, the mAP (%) of the SDD algorithm, and Mask R-CNN algorithm on the gastrointestinal endoscopy image test sample set, the test results are shown in Figure 5.

It can be seen from the experimental results that comparing the SDD algorithm and the Mask R-CNN algorithm, it is found that as the number of training iterations increases for each algorithm, the average accuracy of the detection on the esophageal cancer image test set is also improving but not increase infinitely. That is, for any one of the above three algorithms, the average accuracy mean mAP has an upper limit. Comparing the experimental results of the two algorithms on the esophageal cancer image test sample set at the same number of iterations, the mAP of the SDD algorithm on the esophageal cancer test sample set is better than the mAP of the Mask R-CNN algorithm on the esophageal cancer test sample set.

### 3.2. The Effect of Gastrointestinal Endoscopy Image Verification

As shown in Figure 6, the contrast images of SDD, Mask R-CNN, and manual segmentation of gastrointestinal endoscopy images. Red represents SDD, green represents Mask R-CNN, and yellow represents the effect of manual segmentation. It can be seen from Figure 6 that the red recognition is the most accurate, the manual recognition is the second, and the worst is Mask R-CNN.

## 4. Discussion

Gastrointestinal endoscopic images are the basis for the judgment of gastrointestinal diseases. Due to the complexity of the internal environment, the concealment of pathological features, the blurring of lens shooting, and the complexity of image processing, the occurrence of missed and misdiagnosed phenomena occurs. How to effectively improve the lesion, the real-time performance and accuracy of the detection algorithm is still a more difficult problem. This paper fully understands the current status and challenges of gastrointestinal image lesion detection technology, deeply researches traditional pattern recognition algorithms and deep learning-based target detection algorithms, selects effective algorithms to identify and classify multiple lesions, and achieves efficient detection results.

Lesion detection still faces great challenges, and there are some problems to be solved.

Due to the variable shape and complex texture of gastrointestinal lesions, the number of existing endoscopic pictures is lacking. There are tens of thousands of pictures in a gastrointestinal endoscopy, and few can be used for actual labeling. After screening, an average of 30 can be used for image labeling. The data sets of the three types of lesions constructed in this paper need to be greatly expanded, and the collection of a large number of endoscopic images is a necessary work for further research.

The algorithm in this paper is mainly for single image detection, which cannot meet the real-time detection of video images in practical applications. It is necessary to build a lesion detection system for gastrointestinal endoscopy images and establish a relational database between patients and medical staff.

mAP needs to be improved. Due to the limitations of many factors, the experimental results of this article still have a lot of room for improvement in detection accuracy. The algorithm and network framework need to be further improved, and the weight settings between each network layer are measured to achieve the best detection effect.. The use of convolutional neural networks to extract lesion features requires higher equipment requirements, and the complex network structure will result in slower algorithm processing speed. Therefore, how to improve the processing speed of the algorithm while making full use of the features of the convolutional neural network will be the focus of future research.

This paper makes a preliminary exploration of the deep learning target detection algorithm based on the region of interest on the esophageal cancer image, and further research is needed. At the same time, it is still necessary to study the experimental effects of other deep learning target detection algorithms on esophageal cancer images.

## 5. Conclusion

The mean Average Precision (mAP) of our proposed SSD network is 95.74%, 12.4% higher than manual detection, and 5.7% higher than Mask R-CNN. When detecting a single frame of image, the detection speed of SSD is 8.41 times that of manual detection. We select a variety of algorithms to identify and classify polyps to achieve efficient detection results. It shows that deep learning has a lot of room for development in the field of gastrointestinal image recognition.

## Figures and Tables

**Figure 1:** Polyp detection flowchart of deep learning algorithm.

**Figure 2:** SSD network structure.

**Figure 3:** Mask R-CNN algorithm architecture diagram.

**Figure 4:** mAP of each data set in 6000 iterations.

**Figure 5:** Iterate the mAP of two models of 3000, 6000, 9000, and 12000.

**Figure 6:** Comparison of the effects of three ways to identify polyps.

**Table 1:** Gastrointestinal endoscopy image data set.

Style	Train	Eval	Test
Polyp	1200	800	850
Bleeding	800	700	650
Total	2000	1500	1400

## Data Availability

The image data used to support the findings of this study have been deposited in the Kvasir-SEG data set (https://munin.uit.no/handle/10037/18342).
